# Interleukin‐1 blockade treatment decreasing cardiovascular risk

**DOI:** 10.1002/clc.23246

**Published:** 2019-08-15

**Authors:** Zi‐Heng Zheng, Xun Zeng, Xiao‐Ying Nie, Yun‐Jiu Cheng, Jun Liu, Xiao‐Xiong Lin, Hao Yao, Cheng‐Cheng Ji, Xu‐Miao Chen, Fan Jun, Su‐Hua Wu

**Affiliations:** ^1^ Department of Cardiology The First Affiliated Hospital, Sun Yat‐Sen University and Key Laboratory on Assisted Circulation, NHC Guangzhou China; ^2^ Outpatient Department The First Affiliated Hospital, Sun Yat‐Sen University Guangzhou China

**Keywords:** anakinra, canakinumab, cardiovascular events, Interleukin‐1 blockade, meta‐analysis

## Abstract

**Background:**

Interleukin‐1 (IL‐1) played a role in the occurrence and development of atherosclerosis and cardiovascular events. However, the association between IL‐1 blockage treatment and reducing of cardiovascular risk remains poorly defined.

**Hypothesis:**

IL‐1 blockage treatment reduce the risk and incidence rate of overall major adverse cardiovascular events (MACE), all‐cause death, acute myocardial infarction(MI), unstable angina and heart failure.

**Methods:**

We performed a search of published reports by using MEDLINE database (January 1, 2005 to April 1, 2018). The randomized controlled trials (RCTs) that reported sample size and occurrence numbers in test group and placebo group for the associations of interest were included.

**Results:**

Eight RCT studies involving 15 647 participants were identified. Compared with those who took no IL‐1 blockage, patients taking IL‐1 blockage experienced a decreased risk of overall MACE (RR 0.88, 95% CI 0.82‐0.94), unstable angina (RR 0.80, 95% CI 0.66‐0.98), and breakthrough or recurrence of heart failure (RR 0.44, 95% CI 0.22‐0.87). No association was found between IL‐1 blockage treatment and death from all cause (RR 0.91, 95% CI 0.83‐1.00) as well as acute MI (RR 0.85, 95% CI 0.71‐1.01). The RRs associated with overall MACE, death from all cause, acute MI, and unstable angina for anakinra were 1.05, 1.16, 2.97, and 0.56, respectively, and for canakinumab were 1.05, 0.91, 0.80, and 0.80, respectively.

**Conclusions:**

Administration of IL‐1 blockage was associated with decrease risks of overall MACE, unstable angina, and breakthrough or recurrence of heart failure, but not with death from all cause as well as acute MI.

## 1 INTRODUCTION

A chronic low‐grade inflammatory reaction as an important role in the pathophysiological procedure in the occurrence and development of atherosclerosis and cardiovascular diseases is now largely accepted.^1^, ^2^ Anti‐inflammatory therapy provided a new treatment strategy in some cardiovascular diseases and the secondary prevention of cardiovascular events.^3^, ^4^ There are many inflammatory factors that mediate the process of chronic inflammation. IL‐1 is well known as one of the main members of the inflammatory factor family. The process of inflammation mediated by IL‐1 can cause many kinds of diseases.^5^, ^6^, ^7^ Long‐term chronic inflammation can lead to the formation of arterial plaques as well as atherogenesis,^8^ and active inflammatory process may trigger the rupture of plaque which increasing the risk of coronary thrombosis, then leading to clinical ischemic events.^9^

There are four IL‐1 blockers available now, anakinra, canakinumab, rilonacept, and gevokizumab.^10^, ^11^, ^12^, ^13^ Anakinra is the main kind of IL‐1 blocker. It is a recombinant human IL‐1 receptor antagonist that competitively inhibit IL‐1b and IL‐1a by binding the IL‐1 receptor type I. A number of clinical studies are reported about anakinra used in the treatment of rheumatoid arthritis and approved its effectiveness.^11^, ^12^, ^13^ It was also studies in used of adult‐onset Still,^14^ gout,^15^ Behçet's disease,^16^ and other autoimmune diseases. In an animal experiment with mouse model of AMI, anakinra was given before the surgical induction of Ischemia/reperfusion. The study showed that compared with mice in vehicle‐treated group the mice in anakinra prophylactic treatment group had higher LVEF and less infarct size.^17^ It approved the function of protection of myocardium and preservation of cardiac function using anakinra treatment before the onset of AMI. Other animal experiments were also launched confirming the cardiovascular effectiveness of anakinra.^18^, ^19^ Clinical trials about anakinra's effectiveness on reducing cardiovascular risk and cardiovascular events have also been developed. Canakinumab is a human monoclonal anti‐human IL‐1b antibody that can significantly lower the level of CRP.^20^ Cryopyrin‐associated periodic syndromes, a series of IL‐1b driven inflammatory disorders, have been confirmed that could be induced rapid and sustained remission of symptoms by using canakinumab.^20^, ^21^, ^22^ Other clinical trials also have been launched to confirm the effectiveness on treatment with canakinumab in arthritis, diabetes, and gout patients, and have been shown to lower CRP levels.^23^, ^24^, ^25^ There have been only a few published studies of canakinumab in patients with coronary artery disease. Its effectiveness on cardiovascular diseases still needs more further researches.

Given these backgrounds, we conducted a meta‐analysis to summarize all published RCT studies to examine whether IL‐1 blockage treatment reduce the risk and incidence rate of overall major adverse cardiovascular events, all‐cause death, acute myocardial infarction, unstable angina and heart failure.

## 2 METHODS

The meta‐analysis was conducted following the PRISMA guidelines (Text S1). We performed a systematic search of relevant studies published from January 1, 2005 to April 1, 2018 in the MEDLINE databases with no restrictions.

### 2.1 Search Strategy

The following text and key words in combination: “IL‐1β Inhibition” and “Atherosclerosis,” “cardiovascular,” “myocardial infarction,” “Acute coronary syndrome,” “ACS,” “stroke”; “IL‐1 block” and “Acute coronary syndrome,” “Atherosclerosis,” “cardiovascular,” “ACS,” “stroke,” “myocardial infarction”; “IL‐1 inhibition” and “ACS,” “cardiovascular,” “stroke,” “Acute coronary syndrome,” “myocardial infarction,” “Atherosclerosis”; “canakinumab” and “ACS,” “Acute coronary syndrome,” “Atherosclerosis,” cardiovascular,” “myocardial infarction,” “stroke,” “diabetes”; “anakinra” and “ACS,” “Acute coronary syndrome,” “Atherosclerosis,” “cardiovascular,” “myocardial infarction,” “stroke,” “diabetes” were used to search for studies published from January 1, 2005 to April 1, 2018 in the MEDLINE databases. We manually checked the reference list of each retrieved report to identify other relevant studies in order to identify any studies that were not identified from the preliminary searches.

### 2.2 Study Selection

The following methodological restrictions were imposed for the inclusion criteria to minimize differences between studies: (1) Published in the English language with research method of randomized controlled trials (RCTs), published as original articles. (2) The subjects must have the basis of cardiovascular disease or cardiovascular complications of other diseases can cause cardiovascular disease. (3) The studies must present the sample size, occurrence number and nonoccurrence number both in test group and placebo group of each relevant end point. In instances of multiple publications, the most up to date or comprehensive information was used.

### 2.3 Data Abstraction

From each retrieved report, we extracted the following data: name of the lead investigator, year of publication, country where the study was performed, methods for assessment of end points, main investigational drug the study use, the sample size of the study including total sample size as well as sample size of test group and placebo group, average age of test group and placebo group, proportions of men and women of test group and placebo group, Body Mass Index(BMI) of test group and placebo group, proportions of hypertension patients of test group and placebo group, proportions of diabetes patients of test group and placebo group, mean and mean's 95% Confidence Interval (CI) of C Reactive Protein (CRP) on the baseline of test group and placebo group, end point of each study.

### 2.4 Statistical Analysis

We used Relative Risk (RR) for the measure of the association between IL‐1 blockage treatment and cardiovascular risk. Heterogeneity among studies was formally assessed using Q and I^2^ statistics applying the following interpretation for Q and I^2^: *P* > .1 = low heterogeneity, *P* < .1 = high heterogeneity; I^2^<50% = low heterogeneity, 40% < I^2^ < 60% = moderate heterogeneity, I^2^>60% = high heterogeneity. Fixed‐effects models were used for estimating pooled RRs if heterogeneity among studies was permissible (both *P* > .1 and I^2^ < 40%). When there was biggish heterogeneity among studies (*P* < .1 or I^2^ > 40%), random rather than fixed effects models was used in order to take into account the heterogeneity. Subgroup analyses, meta‐regression models and sensitivity analysis would be carried out to investigate potential sources of between‐study heterogeneity if there was high heterogeneity among studies. Publication bias was tested using funnel plot and Egger's regression test. We used STATA, version 14.0 (Stata Corp LP, College Station, TX) for all analyses. Two‐sided *P* values <.05 were considered statistically significant.

## 3 RESULTS

### 3.1 Study Selection

The results of the search were shown in Figure 1. Five‐hundreds and twenty‐six studies were reviewed in preliminary search. Of these 458 studies were excluded because they were not RCTs. In 68 RCTs with abstract review, there were 51 not‐relevant studies or duplicated studies. Then we read the full review of remaining 17 studies for detailed reading. However, four studies were excluded as not including or not all cardiovascular patients, one was excluded as cross‐over study, one was excluded as not finding full review, two were excluded as results not published yet, one was excluded as cannot be combined for change rates of CRP. The leaving eight studies were finally included in the meta‐analysis.

**Figure 1:** Flowchart of the selection of studies included in meta‐analysis

### 3.2 Study Characteristics

A total of 15 647 individuals were included in eight studies, in which 74.6% were male. The year of publication of these studies ranged from 2010 to 2017. Of those eight studies, eight studied for drug of anakinra and three for canakinumab. All eight studies evaluated the end points of overall major adverse cardiovascular events and death from any cause with Interleukin‐1 blockade treatment, seven studies evaluated the end points of acute myocardial Infarction, six studies evaluated the end points of unstable angina, five studies evaluated the end points of breakthrough or recurrence of heart failure. The detailed data of age, body mass index (BMI), proportion of hypertension, proportion of diabetes, and baseline of patient's C reactive protein (CRP) are showed in Table 1.

**Table 1:** Characteristics of the included eight RCTs

No. of Article	1	2	3	4	5	6	7	8
First author	Benjamin W. Van Tassell	Allison C. Morton	Antonio Abbate	Antonio Abbate	Antonio Abbate	Robin P. Choudhury	P.M. Ridker	P.M. Ridker
Year	2017	2014	2010	2013	2015	2016	2017	2017
Region	America	UK	America	America	America	Canada,UK,America,Germany and Israel	39 Countries	39 Countries
Trial type	RCT	RCT	RCT	RCT	RCT	RCT	RCT	RCT
Drug	Anakinra	Anakinra	Anakinra	Anakinra	Anakinra	Canakinumab	Canakinumab	Canakinumab
Case(n[P/T])	34(18/16)	182(89/93)	10(5/5)	30(15/15)	40(20/20)	189(94/95)	5628(3344/2284)	9534(3182/6352)
Age (P/T)	61(56‐68)/57(53‐66)	61.3(12.3)/61.4(11.7)	51.8(28‐65)/45.4(34‐59)	58.2(35‐83)/59.1(46‐86)	58(51‐65)/57(48‐60)	61.9(6.9)/61.7(7.8)	61.1(10.0)/61.2(10.0)	61.0(54.0‐68.0)/61.0(55.0‐68.0)(T1);61.0(54.0‐68.0)(T2)
Male (n[%]) (P/T)	13(72)/12(75)	67(75.3)/63(67.7)	5(100)/3(60)	13(86.7)/9(60.0)	18(90)/12(60)	80(85)/82(86)	2479(74.1)/1709(74.8)	2365(74)/4735(75)
BMI(kg/㎡)	30(27‐38)/36(29‐41)	28.4(4.7)/30.0(7.1)	NA	NA	NA	30.3(4.0)/30.3(4.1)	NA	29.7(26.6‐33.9)/30.5(27.0‐34.7)(T1);29.6(26.4‐33.1)(T2)
Hypertestion(%) (P/T)	NA	29(32.6)/31 (33.3)	3(60)/5(100)	11(73.3)/7(46.7)	14 (70)/12(60)	83(88)/81(85)	2644(79.1)/1814(79.4)	2514(79)/5075(80)
Diabetes(%)(P/T)	12(67)/9(56)	8(9.0)/15(16.1)	1(20)/2(40)	3(20.0)/3(20.0)	4(20)/5(25)	81(86)/81(85)	1333(39.9)/1814(79.4)	1265(40)/2536(40)
CRP([mg/L])(P/T)	5.2(2.0‐11.9)/7.2(3.3‐12.3)	5.21(3.75, 7.22)/5.38(4.12, 7.04)	NA	4.3(2.2‐7.5)/7.0(2.3‐8.7)	NA	1.85(0.83‐3.88)/1.77(0.84‐3.74)	4.10(2.75‐6.85)/4.25(2.85‐7.05)	4.10(2.75–6.85)/5.55 (3.60‐9.25)(T1);3.40(2.45‐5.20)(T2)
End point	All MACE ALL death AMI UA HF	All MACE ALL death AMI	All MACE ALL death AMI UA HF	All MACE ALL death AMI UA HF	All MACE ALL death AMI UA HF	All MACE ALL death AMI UA HF	All MACE ALL death AMI UA	All MACE ALL death

Abbreviations: AMI, acute myocardial infarction; AUC, area under curve; BMI, body‐mass index; CRP, C reactive protein; HF, heart failure; LVESVi, left ventricular end systolic volume index; MACE, major adverse cardiovascular event; NA, not available; P, placebo group; RCT, randomized controlled trial; T, test group; T1, test group1; T2, test group2; UA, unstable angina.

### 3.3 Association with overall major adverse cardiovascular events

Eight studies reported the outcome of overall major adverse cardiovascular events with 15 467 participants and 2809 events (Figure 2). Overall, using of Interleukin‐1 blockade treatment was associated with a decreased risk of overall major adverse cardiovascular events (RR 0.88, 95% CI 0.82‐0.94) with low between‐study heterogeneity using fixed‐effects model (I^2^: 37.3%, *P* = .131) (Figures 2 and 3). Neither funnel plots (Supplement Figure 1) nor Egger and Begg tests showed evidence of publication bias (Egger, *P* = .763; Begg, *P* = 1.000).

**Figure 2:** Interleukin‐1 Blockade treatment and Cardiovascular Risk. The dotted line in the forest plot represents fixed‐effects summary risk estimate

**Figure 3:** Forest plot showing relative risks of overall major adverse cardiovascular events, death from any cause, acute myocardial Infarction, unstable angina and breakthrough or recurrence of heart failure. The size of each square is proportional to the study's weight (inverse of variance). The dotted line in the forest plot represents fixed‐effects summary risk estimate

In subgroup analysis by investigational drug, using of anakinra shows no association with a decreased or increased risk of overall major adverse cardiovascular events (RR 1.05, 95% CI 0.68‐1.61) with high between‐study heterogeneity using fixed‐effects model (I^2^: 60.0%, *P* = .041) while using of canakinumab shows the association with a decrease risk of overall major adverse cardiovascular events (RR 0.87. 95% CI 0.81‐0.94) with low between‐study heterogeneity using fixed‐effects model (I^2^: 0.0%, *P* = .582) (Figure 4). To explore study heterogeneity between studies of using anakinra, we used the random‐effects model instead of model showing little of risk estimation (RR 0.89, 95% CI 0.41‐1.90) and between‐study heterogeneity (I^2^: 60.0%, *P* = .041). There was a larger sample study that is opposite to the result direction (RR 3.35, 95% CI 1.15‐9.79) (Figure 4). To further explore study heterogeneity, a sensitivity analysis was done to removing this larger sample study with the abnormal result. After removing this study, the result of meta‐analysis with the remaining studies also showing no association with risk of overall major adverse cardiovascular events (RR 0.68, 95% CI 0.42‐1.11) but with low between‐study heterogeneity using fixed‐effects model (I^2^: 20.2%, *P* = .289).

**Figure 4:** Forest plot showing result of by subgroup analysis by investigational drug about relative risks of overall major adverse cardiovascular events, death from any cause, acute myocardial Infarction, unstable angina. The size of each square is proportional to the study's weight (inverse of variance). The dotted line in the forest plot represents fixed‐effects summary risk estimate

### 3.4 Association with death from all cause

Eight studies reported the outcome of death from all cause with 15 467 participants and 1566 events (Figure 2). Overall, using of Interleukin‐1 blockade treatment was associated with no decreased or increased risk of death from all cause (RR 0.91, 95% CI 0.83‐1.00) with low between‐study heterogeneity using fixed‐effects model (I^2^: 0.0%, *P* = .825) (Figure 2 and 3). Neither funnel plots (Supplement Figure 1) nor Egger and Begg tests showed evidence of publication bias (Egger, *P* = .645; Begg, *P* = 1.000).

In subgroup analysis by investigational drug, using of anakinra showed no association with a decreased or increased risk of death from all cause (RR 1.16, 95% CI 0.40‐3.40) with low between‐study heterogeneity using fixed‐effects model (I^2^: 0.0%, *P* = .575) while using of canakinumab also shows no association with a decreased or increased risk of death from all cause (RR 0.91, 95% CI 0.82‐1.00) with low between‐study heterogeneity using fixed‐effects model (I^2^: 0.0%, *P* = .712) **(**Figure 4).

### 3.5 Association with acute myocardial infraction

There were seven studies reporting the outcome of acute myocardial infraction with 6113 participants and 472 events (Figure 2). Overall, using of Interleukin‐1 blockade treatment was associated with no decreased or increased risk of acute myocardial infraction (RR 0.85, 95% CI 0.71‐1.01) with low between‐study heterogeneity using fixed‐effects model (I^2^: 18.4%, *P* = .289) (Figures 2 and 3). However, funnel plots (Supplement Figure 1) and Egger tests showed there was the evidence of publication bias (Egger, *P* = .014). We used trim and fill method for test publication bias. The result showed that there were three studies defecting after four iterations. The pooled effect after trimming and filling (OR 0.88, 95% CI 0.70‐1.06) did not change largely compared with the pooled effect before trimming and filling (OR 0.842, 95% CI 0.662‐1.022). In addition, result of test for heterogeneity also did not change (I^2^: 23.81% before trimming and filling as well as I^2^: 32.19% after trimming and filling). Although there is publication bias, the result is steady.

In subgroup analysis by investigational drug, using of anakinra showed the association with an increased risk of acute myocardial infraction (RR 2.97, 95% CI 1.11‐7.93) with low between‐study heterogeneity using fixed‐effects model (I^2^: 0.0%, *P* = .931) while using of canakinumab shows the association with a decreased risk of acute myocardial infraction (RR 0.80, 95% CI 0.67‐0.97) with low between‐study heterogeneity using fixed‐effects model (I^2^: 0.0%, *P* = .456) using fixed‐effects model (I^2^: 0.0%, *P* = .712) (Figure 4).

### 3.6 Association with unstable angina

There were six studies reporting the outcome of unstable angina with 5931 participants and 460 events (Figure 2). Overall, using of Interleukin‐1 blockade treatment was associated with a decreased risk of unstable angina (RR 0.80, 95% CI 0.66‐0.98) with low between‐study heterogeneity using fixed‐effects model (I^2^: 0.0%, *P* = .819) (Figures 2 and 3). Neither funnel plots (Supplement Figure 1) nor Egger and Begg tests showed evidence of publication bias (Egger, *P* = .979; Begg, *P* = .734).

In subgroup analysis by investigational drug, using of anakinra showed no association with an increased or decreased risk of unstable angina (RR 0.56, 95% CI 0.13‐2.37) with low between‐study heterogeneity using fixed‐effects model (I^2^: 0.0%, *P* = .692) while using of canakinumab shows the association with a decreased risk of unstable angina (RR 0.80, 95% CI 0.67‐0.97) with low between‐study heterogeneity using fixed‐effects model (I^2^: 0.0%, *P* = .456) using fixed‐effects model (I^2^: 0.0%, *P* = .819) (Figure 4).

### 3.7 Association with breakthrough or recurrence of heart failure

Five studies reported the outcome of breakthrough or recurrence of heart failure with 303participants and 31 events (Figure 2). Overall, using of Interleukin‐1 blockade treatment was associated with a decreased risk of breakthrough or recurrence of heart failure (RR 0.44, 95% CI 0.22‐0.87) with low between‐study heterogeneity using fixed‐effects model (I^2^: 13.6%, *P* = .327) (Figures 2 and 3). Neither funnel plots (Supplement Figure 1) nor Egger and Begg tests showed evidence of publication bias (Egger, *P* = .244; Begg, *P* = 1.000).

In subgroup analysis by investigational drug, using of anakinra shows the association with a decreased risk of outcome of breakthrough or recurrence of heart failure (RR 0.44, 95% CI 0.21‐0.88) with low between‐study heterogeneity using fixed‐effects model (I^2^: 35.5%, *P* = .199) (Figure 4).

### 3.8 Association with CRP

In this meta‐analysis, we also extracted the available CRP data in included studies and have done a simple analysis to evaluate the association between interleukin‐1 blockade treatment and level of CRP. The result showed that using of Interleukin‐1 blockade treatment was associated with a significantly decreased level of CRP (SMD ‐0.30, 95% CI –0.51 to –0.09) with low between‐study heterogeneity using fixed‐effects model (I^2^: 0.0%, *P* = .545) (Figure 4).

## 4 DISCUSSION

The present meta‐analysis showed that administration of interleukin‐1 blockers was associated with decrease risks of overall major adverse cardiovascular events, unstable angina, and breakthrough or recurrence of heart failure.

The possible mechanism that interleukin‐1 blockade treatment decreased the risk of cardiovascular events was that it reduced the inflammatory response thereby decreasing the production of inflammatory mediators, especially the CRP. CRP as a widely used as inflammatory marker in clinical settings, it is also has been recognized as an independent predictor of adverse cardiovascular events.^26^ Many studies have reported that the level of CRP is closely related to the occurrence of adverse cardiovascular events.^27^, ^28^, ^29^ The result of this meta‐analysis showed that in the patients using interleukin‐1 blockade treatment, the level of CRP has been significantly decreased. Several studies have reported the effectiveness of interleukin‐1 blocker used in treatment in diabetes. And significant decrease in CRP level could also be observed in these studies.^30^, ^31^, ^32^ Interleukin‐1 blockers may also decrease cardiovascular risk by reducing related diseases that can cause cardiovascular events, but further studies are still warranted to confirm this presumption.

In the present meta‐analysis, we found that there was no significant association between interleukin‐1 blockade treatment and death from all cause as well as acute myocardial infraction. The one of reasons may be that Infection is a common adverse reaction of interleukin‐1 blockers. Compared with canakinumab, anakinra has the higher risk of Infection owing to inhibit both L‐1b and IL‐1a, especially in patients using immunosuppressive agents at the same time. Clinical studies showed that although the increase of infection‐related deaths was not observed, using anakinra has been associated with an increase in serious infections in patients who were also receiving other immunomodulating agents.^13^, ^33^ Second, patients taking interleukin‐1 blockers might be sicker and have other related diseases like diabetes or gout comparing with patients not taking interleukin‐1 blockers, which can increase the risk of patients' death. Therefore, long‐term survival effect after interleukin‐1 blockade treatment still needs further clinical studies.

There were some limitations to this meta‐analysis. First, when we evaluated the association between anakinra and overall major adverse cardiovascular events, we found there was high between‐study heterogeneity. Sensitivity analysis showed that heterogeneity main came from a larger sample study with an opposite result direction. Second, there was publication bias when evaluating the association with acute myocardial infraction, although trimming and filling showed the result was still steady. Third, the relatively small number of studies limited our ability to compare the risk for reported events between different investigational drugs, especially canakinumab. Fourth, some studies with big sample size and some with small sample size, these big sample size studies showed a greater impact on the trend of results.

Strengths of this study included small between‐studies heterogeneity, long durations of follow‐up and all well‐established clinical RCTs. In addition, our pooled estimates were based on detailed adjustment for confounding variables.

## 5 CONCLUSIONS

In conclusion, the results from our meta‐analysis of clinical RCTs suggested thatinterleukin‐1 blockade treatment was associated with decrease risk of overall major adverse cardiovascular events, unstable angina, and breakthrough or recurrence of heart failure, but not with death from all cause as well as acute myocardial infraction. Future clinical and experimental studies should focus on understanding the exact mechanisms and risk between interleukin‐1 mediated inflammation and cardiovascular events. In addition, large well‐designed RCTs to further evaluate interleukin‐1 blockers' safety and stability of cardiovascular effect are also still needed.

## AUTHOR CONTRIBUTIONS

S.H.W. conceived and designed the experiments. Z.H.Z., X.Z., X.Y.N., Y.J.C., J.L., X.X.L., H.Y., C.C.J., X.M.C., and J.F. performed the experiments. Z.H.Z., X.Z., X.Y.N., Y.J.C., J.L., X.X.L., H.Y., C.C.J., X.M.C., and J.F. analyzed the data. Z.H.Z., X.Z., X.Y.N., Y.J.C., J.L., X.X.L., H.Y., C.C.J., X.M.C., and J.F. contributed reagents/materials/analysis tools. Z.H.Z., X.Z., and X.Y.N. wrote the first draft of the manuscript. Z.H.Z., S.H.W., X.Z., X.Y.N. contributed to the writing of the manuscript. S.H.W., Z.H.Z., X.Z., X.Y.N., Y.J.C., J.L., X.X.L., H.Y., C.C.J., X.M.C., and J.F. read and met ICMJE criteria for authorship. S.H.W., Z.H.Z., X.Z., X.Y.N., Y.J.C., J.L., X.X.L., H.Y., C.C.J., X.M.C., and J.F. agreed with manuscript results and conclusions.

## ETHICS STATEMENT

This study was conducted with the consent of the ethics committee of the first affiliated hospital of Sun Yat‐Sen University. All authors agree the Consent for publication.

## Supporting information


**Supplement Figure 1** Funnel plots showing association of Interleukin‐1 blockade treatment with cardiovascular risk. The horizontal line in the funnel plot indicates the fixed‐effects summary estimate, while the sloping lines indicate the expected 95% confidence intervals for a given SE, assuming no heterogeneity between studies. Symmetrical distribution of circles below and above the horizontal line indicates no evidence of publication bias.

**Text S1** PRISMA 2009 checklist
